# Curcumin Improves Pulmonary Hypertension Rats by Regulating Mitochondrial Function

**DOI:** 10.1155/2021/1078019

**Published:** 2021-08-26

**Authors:** Jing Chen, Wen Jiang, Fei Zhu, Qiong Wang, Haiyan Yang, Jinhua Wu

**Affiliations:** ^1^Department of Pharmaceutics, Zhoushan Women and Children Hospital, 316000, Zhoushan, Zhejiang Province, China; ^2^Department of Teaching & Research, Zhoushan Women and Children Hospital, 316000, Zhoushan, Zhejiang Province, China; ^3^Department of Internal Medicine, Zhoushan Women and Children Hospital, 316000, Zhoushan, Zhejiang Province, China

## Abstract

**Objective:**

To investigate the role of curcumin in regulating pathogenesis of pulmonary arterial smooth muscle cells (PASMCs) derived from pulmonary arterial hypertension (PAH) model.

**Methods:**

Male Sprague Dawley rats were injected with monocrotaline (MCT) to establish the PAH experimental model. The rats were divided into control group, MCT group, and curcumin group. At the end of the study, hemodynamic data were measured to determine pulmonary hypertension. Proliferation ability of PASMCs, a remodeling indicator of pulmonary artery and right ventricle, was detected. In addition, the morphology and function of mitochondria, antiglycolysis and antiproliferation pathways, and genes were also analyzed.

**Results:**

Curcumin may function by reversing MCT-mediated pulmonary vascular remodeling in rats. Curcumin effectively improved pulmonary vascular remodeling, promoted PASMC apoptosis, and protected mitochondrial function. In addition, curcumin treatment suppressed the PI3K/AKT pathway in PASMCs and regulated the expression of antiproliferative genes.

**Conclusion:**

Curcumin can improve energy metabolism and reverse the process of PAHS. However, there were side effects of curcumin in MCT-induced rats, suggesting that the dosage should be treated with caution and its toxicological mechanism should be further studied and evaluated.

## 1. Introduction

Pulmonary arterial hypertension (PAH) is determined by alterations of pulmonary vascular function and structure caused by a variety of factors, leading to a progressive increase in pulmonary vascular resistance. Subsequently, it leads to a clinicopathological syndrome characterized by right ventricular remodeling and right heart failure [1]. The prevalence rate of PAH of all kinds has exceeded 30~50 per 1 million people, making it one of the most important diseases endangering human beings [2]. Despite the improvement of modern drugs and treatment methods, the prognosis of PAH patients is still poor, and the annual mortality rate of 2.5% for females and 0.9% for males has been maintained in the past ten years [3]. Current studies have shown that the degree of increased pulmonary artery pressure is only moderately correlated with clinical prognosis. The functional state of the right ventricle is an independent predictor of clinical symptoms and survival prognosis [4, 5]. Clinical studies have confirmed that different patients show significantly different right ventricular adaptive response and clinical prognosis in response to the same pulmonary vascular resistance [6]. Therefore, it is of great clinical significance to maintain effective right ventricular structure and function. At present, the clinical understanding of right ventricular remodeling mechanism and drug therapy is mainly derived from the left ventricle. Surprisingly, classic drugs that inhibit left ventricular remodeling and left heart failure cannot effectively improve or reverse the right ventricular function and improve the survival rate in PAH patients [7]. It suggests that there are still other mechanisms for right ventricular remodeling and occurrence and development of heart failure. Unfortunately, there is still a lack of an effective and recognized right ventricular specific treatment strategy in clinical practice [8], which is mainly due to the long-term neglect of the importance of right ventricular in PAH course development and the incomplete clarification of the exact mechanism of PAH right ventricular remodeling. An in-depth study of the cellular and molecular mechanisms of PAH right ventricular remodeling has important scientific significance and clinical value for the prevention and treatment of right heart failure and the reversal of functions [9].

Mitochondria are the “power factories” of cells, providing 80% of the energy needed for cell life and play an important role in cell metabolism and physiological processes. It is worth noting that basically all PAH pathological processes seem to be unrelated, and molecules with abnormal expression can be explained by abnormal mitochondrial function. Only cell proliferation and apoptosis are balanced to maintain normal biologic states, while the mitochondria of PAH patients exhibited an antiapoptotic and overproliferative effect in pulmonary artery smooth muscle cell (PASMC), leading to pulmonary vascular remodeling. At the same time, PASMC of PAH patients is also enhanced in the condition of constant oxygen, and mitochondrial function is inhibited, which are strikingly similar to tumor cells [10]. In addition, when PAH occurs, there are molecular markers of tumor cells on the blood vessels, which have been proved to play an important role in the pathological process of PAH [11]. More and more studies have found that various pathological manifestations of PAHS can be explained by the metabolic theory originally used for tumors, and mitochondrial abnormalities are the core of this theory [12]. PASMC also has the characteristic of enhanced glycolysis reaction of tumor cells. Pyruvate dehydrogenase kinase (PDK) plays an important role in PAH generation. PDK prevents pyruvate from entering mitochondria to participate in the Krebs cycle, and insufficient electron production in mitochondrial electron transport chain results in reduced mROS production [13]. At the same time, enhanced glycolysis also promoted pyruvate synthesis of amino acids needed for excessive cell proliferation in the cytoplasm. This mechanism was beneficial to overproliferated cells and promoted pulmonary vascular remodeling.

Curcumin is a kind of fat-soluble phenolic pigment extracted from the traditional Chinese medicine curcuma, which is widely used as food additive. A large number of studies have shown that curcumin has anti-inflammatory, antioxidant, antiviral, scavenging oxygen free radicals, antifibrosis, anticoagulation, lipid regulation, and other pharmacological effects. Curcumin has been paid more and more attention by medical workers at home and abroad because of its low toxicity and good safety [14–16]. Curcumin can significantly reduce aortic injury and neovascularization thickness. Curcumin reduces the expression of CD36 circulating inflammatory factors (IL-1, TNF-*α*, and CRP), intracellular adhesion molecules, vascular cell adhesion molecules, P-selectivity, monocyte chemoattractant protein 1, and mRNA induced by high-fat diet. The study found that low-density lipoprotein gene knockout mice significantly improved early atherosclerosis lesions and lipid exudation in the aortic arch after 18 weeks of long-term curcumin feeding. Curcumin reduces plasma lipid levels, including apolipoprotein B and cholesterol ester transfer protein, and increases the expression of high-density lipoprotein and liver apolipoprotein A1 [17]. Chen et al. investigated the potential effect of curcumin on hypertrophy of cardiomyocytes and the possible mechanism, and the results showed that curcumin inhibited hyperglycemic and insulin-induced cardiac hypertrophy through the PPAR/AKT/NO signaling pathway [18]. In addition, curcumin has other pharmacological effects, such as antifibrosis, neuroprotective effect, promoting wound healing, and reversing multidrug resistance (MDR) of cancer cells. Wang et al. showed that intraperitoneal injection of curcumin could significantly reduce bleomycin-induced pulmonary inflammation and fibrosis response [19]. The mechanism was that curcumin could effectively reduce normal lung tissue and primary pulmonary fibrosis and fibrosis promoting factors and reduce collagen deposition by inhibiting transforming growth factor B. However, the regulation mechanism of curcumin on pulmonary hypertension is still unclear.

It has not been reported whether curcumin inhibits HPA through improving mitochondrial metabolism in hypoxia-induced pulmonary hypertension (HPH) disease model. In this study, through the establishment of HPA rat model and hypoxia PASMC model, the effect mechanism of curcumin on HPA through the regulation of mitochondrial pathway was explored. The purpose of this study was to investigate the role of curcumin in regulating PASMC proliferation and apoptosis, so as to reverse PAH by improving mitochondrial metabolism. This may contribute to the clinical application of curcumin as a new therapeutic agent.

## 2. Methods

### 2.1. Grouping and Treatment of Experimental Animals

Eighteen male SD rats were randomly divided into three groups: normal control group, MCT group, and curcumin group (30 mg·kg^−1^) administrated by gavage. MCT was given with 50 mg·kg^−1^ by subcutaneous injection in one time to prepare the rat pulmonary hypertension model. The animals were given the same dose of saline once a day for 18 consecutive days in the normal group and the model group, and their weight was recorded daily.

The end point was 25 days. The animals were anesthetized with isoflurane and fixed, and the relevant physiological and biochemical indexes such as hemodynamics, organ index, pulmonary inflammatory factors, and immunohistochemistry were measured. For separating and building of rat endothelial cell line, the SD rats were disinfected and anesthetized, and their lung small arteries were isolated from the lung tissues and then treated with 1 mL 0.2% collagenase digestion. I treat lung small artery after digestion of floc centrifugal fragments, to the upper collagenase after joining medium placed at 37°C and 5% CO_2_ cultivation in the box. PASMCs of primary generation were obtained after 3 days, and cells were collected for experiment after cell passage to 4~6 generations. Cell starvation for 12 h synchronizes the cell cycle, followed by intervention.

### 2.2. Cell Activity Was Detected by CCK-8

PASMCs were prepared into single-cell suspension and inoculated into 96-well plates, incubated in a constant temperature incubator for 24 h. The grouping method was the same as before. Each group had 6 holes, and blank groups without cells were set around them, and the corresponding incubator was placed for culture. At the end of the intervention, the medium and CCK-8 reagent are added to each well, and the medium is placed in the incubator in a short time to avoid light, and the absorbance of each hole is set at 450 nm after 1~2 h.

### 2.3. Pulmonary Artery Pressure and Right Cardiac Hypertrophy Measurement

SD rats were anesthetized with isoflurane, and the right external jugular vein was separated after fixation, and the pressure tube was intubated into the pulmonary artery. The mean pulmonary artery pressure (mPAP) of every rat was measured by the physiological recorder [6]. Rats were bleeding to death, and full heart is removed, a complete separation of the right ventricle (right ventricle, RV) and left ventricle and the interventricular septum (left ventricle plus septum, LV + *S*). After being drained and weighed, the right cardiac hypertrophy index (RVHI) = [RV/(LV + *S*)] was recorded and calculated to reflect the condition of right cardiac hypertrophy.

### 2.4. Detection of Pulmonary Vascular Remodeling Index

The upper lobe of the right lung of rats was fixed in 4% paraformaldehyde for 24 h, and the lung tissues were embedded in paraffin for HE staining. The prepared HE staining sections were observed under a common light microscope, and the small pulmonary arteries in 6 different visual fields were randomly selected to be photographed. The Image-pro Plus 6.0 Image analysis software was used to analyze the wall area to total area (WA/TA) of small and medium-sized pulmonary arteries to reflect the degree of pulmonary vascular structural remodeling.

### 2.5. Histological Morphology of Pulmonary Artery Was Determined by HE Staining

The left lung tissue of the rats was fixed on the foam board, and the lung tissue was cut with a scalpel 0.5 cm away from the tip of the lung, and the tissue was fixed in neutral formaldehyde for 24 h. After the tissue was removed, the rats were dehydrated with ethanol, embedded in paraffin, and sliced, and then, HE staining was performed. The pulmonary vascular morphology of each group was observed under an optical microscope. In addition, pulmonary artery with a diameter of about 100 *μ*m was used for quantitative analysis of its morphology using the image analysis software. The ratio of the transection area of the vessel wall to the transection area of the vessel was used as an indicator to measure the remodeling of hypoxic pulmonary vessels.

### 2.6. Immunohistochemical Method Was Used to Detect Ki67 and Apoptosis-Related Proteins Bax and Caspase-3

The left lung tissue of the rats was fixed on the foam board with a pin, and the lung tissue was cut 0.5 cm from the tip of the lung with a scalpel. The pulmonary artery with a diameter of 100 m was isolated and exhaled. The pulmonary artery was fixed with 4% paraformaldehyde and embedded in paraffin, and sections with a thickness of 5 m were prepared for immunohistochemical staining. The slices were dewaxed, followed by the addition of primary antibody at 4°C overnight, followed by the addition of secondary antibody, and dehydrated to seal the slices. The number of positive cells of Ki67, Bax, and caspase-3 in 5 different fields was observed under an optical microscope and then analyzed statistically.

### 2.7. Detection of ATP Content

The tissue was made into 10% homogenate and centrifuged at 2000 × g for 10 min. The supernatant was centrifuged at 1000 × g for 15 min, and the protein was quantified by the Lowry method. The isolated mitochondria were made into suspension with cold homogenate medium, and the contents of ATP were determined.

### 2.8. Preparation of Electron Microscope Samples

The mice in each group were fixed by heart perfusion with 4% glutaraldehyde. The mice were quickly taken out and cut into 1 mm^3^ small pieces and fixed in 4% glutaraldehyde electron microscope solution. According to the preparation procedure of electron microscope samples, the mice were rinsed, dehydrated, soaked, and embedded in epoxy resin. After ultrathin sections, the slices were fished to the copper net and then dried for lead and uranium double staining. The alterations of cell morphology and ultrastructure were observed under transmission electron microscope.

### 2.9. Serum LDH Level Detection

1 ml mouse blood was obtained by eyeball blood sampling method, centrifuged at 3000 × g for 15 min, and the supernatant was stored in -80°C refrigerator. Serum LDH levels were analyzed by enzyme-linked immunosorbent assay (Roche company). The specific operation was carried out in strict accordance with the instructions of the kit. The OD value of 450 nm was recorded for drawing the standard curve and calculating the level of the sample to be measured.

### 2.10. Western Blot Was Used to Detect Protein Expression

Total protein of lung tissue samples and PASMCs was extracted from each group, and the total protein concentration was determined. 40 g cell protein samples and 60 g tissue protein samples were subjected to gel electrophoresis, transferred to PVDF membrane, sealed with skim milk, and incubated at 4°C overnight for primary antibody including p-AKT (abcam,1/1000) and p-PI3K (abcam, 1/1000). Incubate the secondary antibody after washing the next day, and run the imager for exposure after rinsing. Quantity One was used to determine the gray value of each strip, and GAPDH was taken as the internal reference. The ratio of the gray value of proteins in each group to the corresponding GAPDH was the relative expression quantity of the histone, and the expression difference of proteins in each group was compared.

### 2.11. Real-Time PCR (RT-PCR)

Total cellular RNA was extracted using TRIzol and preserved in a -80°C refrigerator. The extracted RNA was subjected to reverse transcription using a cDNA first-strand synthesis kit (TaKaRa, PrimeScript RT Master Mix, RR036A). The reverse transcription synthesis was performed at 37°C for 15 min and 85°C for 5 s and finally preserved at 4°C. PCR amplification of the target genes and the internal reference GAPDH was carried out using SYBR Premix Ex Taq II, RR820A (Takara, Dalian, China). Primer sequences of PKM2 were as follows: forward: 5′-CTCTCACAGTTGAATGTCCTTG-3′ and reverse: 5′-CTCCTTGTCAGCAGAATGAAG-3′. Primer sequences of MCT1 were as follows: forward: 5′-AGAAGGCTGGGGCTCATTTG-3′ and reverse: 5′-AGGGGCCATCCACAGTCTTC-3′. Primer sequences of PTEN were as follows: forward: 5′-CTCTCACAGTTGAATGTCCTTG-3′ and reverse: 5′-ATCCGGTCAGCAGAATGAAG-3′. Primer sequences of SRC were as follows: forward: 5′-GGTCAATCGGCTCATTTG-3′ and reverse: 5′-GTGTCCATCCACAGTCTTC-3′. RT-PCR was conducted at 95°C for 30 s, 95°C for 5 s, and 60°C for 30 s, for a total of 40 cycles. Expression level of target gene was calculated by the 2–*ΔΔ*Ct method.

### 2.12. Statistical Analysis

The difference of indicators between 3 groups was analyzed by *t*-test and *P* < 0.05 indicated that the difference was statistically significant. The SPSS21.0 statistical software was used for analysis. Multigroup comparisons were performed by one-way ANOVA, and pairwise comparisons were performed by the LSD-t method.

## 3. Results

### 3.1. Curcumin Improves Vascular Remodeling

Right ventricular systolic pressure (RVSP) and mean pulmonary arterial pressure (mPAP) were significantly raised in MCT-induced rats but decreased after curcumin administration (Figures 1(a) and 1(b)). Furthermore, MCT-mediated pulmonary arterioles were observably remodeled. However, after curcumin delivery, this influence was significantly reduced by increasing the mean median thickness, lumen/total ratio, and pulmonary WT% (*P* < 0.05) as shown in Figures 1(c)–1(f). These results illustrate that curcumin may function by reversing MCT-mediated pulmonary vascular remodeling in rats.

### 3.2. Curcumin Can Improve Ventricular Function

Compared with the control group, RVHI in MCT group was observably higher but decreased after curcumin delivery (Figure 2(a)). In addition, after curcumin delivery, RV fibrosis was also uniformly reversed. In the MCT group, RV fibrosis was boosted compared with the control group, while curcumin group was reversed (Figure 2(b)). Of note, RV thickness and interventricular septum diameter (IVSD) boosted in the MCT group but decreased in the curcumin group (*P* < 0.05), as shown in Figures 2(c) and 2(d). Tricuspid annular plane systolic excursion (TAPSE), an indicator of RV systolic function, also improved after curcumin delivery. Compared with the control group, TAPSE decreased in the MCT group and boosted in the curcumin group (Figure 2(e)). Therefore, our results suggested that curcumin normalizes right ventricular function by reducing pulmonary artery pressure.

### 3.3. Curcumin Promotes Apoptosis of PASMC

To evaluate the influence of curcumin on PASMC proliferation, lung tissue sections were stained. The percentage of Ki67 positive cells around pulmonary artery in the MCT group was significantly boosted. However, this influence was reversed after curcumin administration (*P* < 0.05; Figure 3(a)). To further confirm the involved influence, PASMCs were isolated from all three groups for culture. The OD value of the MCT group was higher than that of the control group, while that of the curcumin group was lower than that of the MCT group (*P* < 0.05; Figure 3(b)), suggesting curcumin inhibited the proliferation of PASMC in PAH rat models.

In addition, lung tissue sections were stained to detect apoptotic markers Bax and caspase-3. Compared with the control group, the percentage of Bax and caspase-3 positive cells in the MCT group diminished, while that in the curcumin group triggered (both *P* < 0.05) as shown in Figures 3(c) and 3(d). Therefore, curcumin can markedly promote the apoptosis of PASMC in MCT-mediated PAH models.

### 3.4. Curcumin Improves Function of Mitochondrial

Morphological analysis showed that compared with the control group, MCT administration markedly reduced the number of normal mitochondria and triggered the number of mitochondrial fragments. After curcumin administration, the influence was weakened (Figures 4(a) and 4(b)). To assess mitochondrial function, ATP content in lung tissue was measured. The results showed that the ATP level in the MCT group was lower than that in the control group. However, the curcumin group triggered compared with the MCT group (Figure 4(c)). Serum LDH concentration was measured to further reflect the metabolic state. LDH in the MCT group was boosted compared with that in the control group, while that in the curcumin group was decreased (Figure 4(d)) and showed that curcumin markedly protected mitochondrial functions in MCT-induced PAH rat models.

### 3.5. Curcumin Inhibits the PI3K/AKT Pathway in PASMCs

Next, we investigated whether curcumin mediates the proliferation and apoptosis of PASMC by hindering the PI3K/AKT pathway. Compared with the control group, the expression of p-PI3K and p-AKT was augmented in the MCT group (*P* < 0.05). Compared with the MCT group, the expression of p-PI3K and p-AKT in the curcumin group was decreased (all *P* < 0.05; Figure 5(a)). These findings illustrate the curcumin PASMC proliferation inhibition by PI3K/AKT pathway.

### 3.6. Curcumin Mediated the Expression of Antiproliferative Genes in PASMCs

Compared with the control group, the relative expressions of PKM2, MCT1, and SRC in the MCT group were augmented, respectively, while PTEN was diminished (all *P* < 0.05). After curcumin administration, the protein levels of PKM2, MCT1, and SRC were suppressed while PTEN were diminished, respectively, compared with the MCT group (*P* < 0.05; Figures 5(b)–5(f)). These results indicated that curcumin could significantly induce the expression of antiglycolysis and antiproliferation genes in PASMCs.

## 4. Discussion

Changing the imbalance of proliferation/apoptosis of smooth muscle and endothelial cells has long been a key strategy to prevent vascular remodeling. There is evidence that promoting smooth muscle cell apoptosis under hypoxic exposure, such as artificially induced expression of smooth muscle cell tumor suppressor gene P27, can effectively improve vascular remodeling [20]. However, after administration of a broad-spectrum inhibitor of caspase-3 in rats, hypoxia-induced apoptosis of endothelial cells was reduced and hypoxia-induced pulmonary vascular remodeling was significantly inhibited. Apoptosis of smooth muscle cells is involved in the reversal process of vascular remodeling. In the process of reoxygenation, the production of reactive oxygen species in cells increases and mediates cell apoptosis. After the removal of reactive oxygen species, its apoptosis can be significantly inhibited [20, 21]. Other pathways including activation of P53, inhibition of STAT3 pathway, inhibition of mitochondrial division, activation of autophagy, and inhibition of NLRP3 inflammasome activation can all inhibit hypoxia-induced smooth muscle cell proliferation and endothelial cell injury and improve vascular remodeling [22].

Herein, we demonstrate that curcumin significantly reduces pulmonary vascular remodeling in the rat model of pulmonary hypertension. Another recent study showed that curcumin treatment significantly restored mitochondrial structure, thereby inhibiting PAHs. Notably, we demonstrate that curcumin can improve mitochondrial metabolism, inhibit PASMC proliferation, promote apoptosis, and ultimately reduce pulmonary vascular remodeling and RV dysfunction. In addition, we found that curcumin plays a protective role in PAH by inhibiting the PI3K/AKT pathway. In terms of molecular mechanism, curcumin treatment attenuates the expression of antiglycolysis and antiproliferation genes mediated by MCT treatment.

In recent years, mitochondria have attracted much attention as a research hotspot. Mitochondria not only serve as an energy factory, but also as a transfer station for the collection and transmission of various intracellular signals, which are widely involved in cell autophagy, inflammatory response, proliferation/apoptosis, and other cellular biological processes. Under hypoxic exposure, the mitochondrial structure and function of endothelial cells and smooth muscle cells were abnormally changed. Smooth muscle cells in vascular remodeling exhibit malignant proliferation similar to cancer cells. Even in the presence of sufficient oxygen, mitochondrial aerobic oxidation is inhibited and glycolytic metabolism is enhanced. Mitochondrial membrane potential and mitochondrial oxygen free radical were also changed. A series of abnormalities in mitochondria can activate downstream-related pathways, thereby activating the transcription of proliferation-related genes and promoting cell proliferation [23, 24]. Reduced concentration of mitochondrial calcium can inhibit the activity of Ca2+-dependent enzymes in mitochondria, including pyruvate dehydrogenase (PDH), isocitrate dehydrogenase, *α*-ketoglutarate dehydrogenase, and ATP synthase, which inhibit glucose oxidation and promote glycolysis. The reduction of the intermediate *α*-ketoglutarate (*α*-KG) and mitochondrial oxygen free radicals relieved the inhibition of HIF prolyl hydroxylase and inhibited the activity of P53, thereby activating HIF-1*α* at the transcription and protein levels. At the same time, HIF-1*α* inhibits mitochondrial biosynsis and promotes the expression of glycosylated enzymes such as pyruvate dehydrogenase kinase (PDK), which phosphorylates PDH, thus forming a positive feedback regulation of amplification and further promoting smooth muscle cell proliferation. In another key cell of vascular remodeling, hypoxia can cause mitochondrial crista fracture and swelling in endothelial cells and also activate mitochondrial autophagy, damaging mitochondrial biosynthetic [25–27], which leads to endothelial cell damage, activation of the NF-*κ*B pathway-mediated inflammatory molecule expression, inhibition of NO production, and promotion of contractibility factor secretion.

As for PHA-related research fields, it has been reported that caspase-1 can regulate inflammatory factors and participate in the occurrence and development of PHA [28]. IL-1 can mediate the recruitment of macrophages around pulmonary vessels in mice, promote the abnormal proliferation of PASMCs, and cause pulmonary vascular remodeling, which is closely related to the disease progression of PHA [29, 30]. Curcumin could inhibit the secretion of IL-1 by inhibiting NLRP3 inflammasome, thus playing an anti-inflammatory role. Since inflammation is one of the important pathological mechanisms of hypoxia injury, curcumin may inhibit the activation of caspase-1 by inhibiting NLRP3 inflammasome, thereby reducing the maturation and release of IL-1, reducing the proliferation of inflammation-induced PASMCs, improving the remodeling of blood vessels, and ultimately reducing pulmonary artery pressure in PHA rats.

## 5. Conclusion

Pulmonary hypertension is a serious disease characterized by pulmonary vascular structure and remodeling, right heart failure, and eventual death. Mitochondrial metabolic changes have recently been recognized as a new feature of PAH. Therefore, correcting mitochondrial metabolism can inhibit the excessive proliferation of PASMCs and promote its apoptosis, which is the core mechanism of PAH. Our results show that curcumin can reduce pulmonary artery pressure and remodeling, so it may be a new drug for PAH. Overall, our data suggest that curcumin is effective in reducing pulmonary artery pressure and reversing pulmonary artery remodeling but should be used with caution.

## Figures and Tables

**Figure 1:** Curcumin improves vascular remodeling. (a) Data results of RVSP (mmHg). (b) Data results of mPAP. (c) Images of HE-stained sections from indicated groups. (d) Data results of artery media thickness. (e) Statistical analysis of pulmonary arterial wall thickness. (f) Data results of lumen of total ratio. ^∗^*P* < 0.05 and ^∗∗^*P* < 0.01. Magnification: 400x.

**Figure 2:** Curcumin can improve ventricular function. (a) RVHI was the ratio of RV weight to LV + *S* weight, RV was stained with picrosirius red and analyzed. (b) Data results of RV fibrosis. (c) Data results of RV wall thickness. (d) Statistical analysis of IVSD. (e) Data results of apical four chamber notch. ^∗^*P* < 0.05 and ^∗∗^*P* < 0.01.

**Figure 3:** Curcumin promotes apoptosis of PASMC. (a) Quantitative analysis of Ki67 positive rate of immunohistochemical staining. (b) The OD value of PASMCs was quantitatively analyzed. (c) Quantitative analysis of the positive rate of Bax. (d) Quantitative analysis of caspase-3 positive rate. ^∗^*P* < 0.05 and ^∗∗^*P* < 0.01.

**Figure 4:** Curcumin improves function of mitochondrial. (a) Statistical analysis of normal mitochondrial percent of RV. (b) Statistical analysis of mitochondrial fragment percent of RV. (c) Effect of curcumin on mitochondrial function in vivo study. Statistical analysis of relative ATP levels in lung tissue. (d) Effect of curcumin on serum LDH concentration. ^∗^*P* < 0.05 and ^∗∗^*P* < 0.01.

**Figure 5:** Curcumin mediated the expression of antiproliferative genes in PASMCs. (a) Relative expression of p-PI3K and p-AKT. (b) Relative expression of PKM2, MCT1, PTEN, and SRC. (c) Quantitative analysis of relative expression of PKM2. (d) Quantitative analysis of relative expression of MCT1. (e) Quantitative analysis of relative expression of PTEN. (f) Quantitative analysis of relative expression of SRC. ^∗^*P* < 0.05 and ^∗∗^*P* < 0.01.

## Data Availability

The data used during the present study are available from the corresponding author upon reasonable request.
